The article "Leukocyte telomere dynamics across gestation in uncomplicated pregnancies and associations with stress" was published in 2022. Journal: BMC Pregnancy Childbirth.

# Leukocyte telomere dynamics across gestation in uncomplicated pregnancies and associations with stress

**DOI:** 10.1186/s12884-022-04693-0

**Published:** 2022-05-02

**Authors:** Danielle M. Panelli, Stephanie A. Leonard, Ronald J. Wong, Martin Becker, Jonathan A. Mayo, Erica Wu, Anna I. Girsen, Ian H. Gotlib, Nima Aghaeepour, Maurice L. Druzin, Gary M. Shaw, David K. Stevenson, Katherine Bianco

**Affiliations:** 1 Department of Obstetrics and Gynecology, Stanford University, 453 Quarry Road, Palo Alto, CA 94304 USA; 2 Department of Pediatrics, Stanford University, Stanford, CA USA; 3 Department of Anesthesiology, Perioperative, and Pain Medicine, Stanford University, Stanford, CA USA; 4 Department of Biomedical Data Science, Stanford University, Stanford, CA USA; 5 Department of Psychology, Stanford University, Stanford, CA USA

**Keywords:** Leukocyte telomere length, Maternal mental health, Psychosocial stress, Pregnancy, Sleep

## Abstract

**Background:**

Short leukocyte telomere length is a biomarker associated with stress and morbidity in non-pregnant adults. Little is known, however, about maternal telomere dynamics in pregnancy. To address this, we examined changes in maternal leukocyte telomere length (LTL) during uncomplicated pregnancies and explored correlations with perceived stress.

**Methods:**

In this pilot study, maternal LTL was measured in blood collected from nulliparas who delivered live, term, singleton infants between 2012 and 2018 at a single institution. Participants were excluded if they had diabetes or hypertensive disease. Samples were collected over the course of pregnancy and divided into three time periods: < 20^0/7^ weeks (Timepoint 1); 20^1/7^ to 36^6/7^ weeks (Timepoint 2); and 37^0/7^ to 9-weeks postpartum (Timepoint 3). All participants also completed a survey assessing a multivariate profile of perceived stress at the time of enrollment in the first trimester. LTL was measured using quantitative polymerase chain reaction (PCR). Wilcoxon signed-rank tests were used to compare LTL differences within participants across all timepoint intervals. To determine whether mode of delivery affected LTL, we compared postpartum Timepoint 3 LTLs between participants who had vaginal versus cesarean birth. Secondarily, we evaluated the association of the assessed multivariate stress profile and LTL using machine learning analysis.

**Results:**

A total of 115 samples from 46 patients were analyzed. LTL (mean ± SD), expressed as telomere to single copy gene (T/S) ratios, were: 1.15 ± 0.26, 1.13 ± 0.23, and 1.07 ± 0.21 for Timepoints 1, 2, and 3, respectively. There were no significant differences in LTL between Timepoints 1 and 2 (LTL T/S change − 0.03 ± 0.26, *p* = 0.39); 2 and 3 (− 0.07 ± 0.29, *p* = 0.38) or Timepoints 1 and 3 (− 0.07 ± 0.21, *p* = 0.06). Participants who underwent cesareans had significantly shorter postpartum LTLs than those who delivered vaginally (T/S ratio: 0.94 ± 0.12 cesarean versus 1.12 ± 0.21 vaginal, *p* = 0.01). In secondary analysis, poor sleep quality was the main stress construct associated with shorter Timepoint 1 LTLs (*p* = 0.02) and shorter mean LTLs (*p* = 0.03).

**Conclusions:**

In this cohort of healthy pregnancies, maternal LTLs did not significantly change across gestation and postpartum LTLs were shorter after cesarean than after vaginal birth. Significant associations between sleep quality and short LTLs warrant further investigation.

**Supplementary Information:**

The online version contains supplementary material available at 10.1186/s12884-022-04693-0.

## Background

Leukocyte telomere length (LTL) is a biomarker associated with increased morbidity and mortality in non-pregnant adults; however, little is known regarding maternal LTL during pregnancy. Over one’s lifespan, LTL shortens continuously, with medical and psychological stressors accelerating the shortening rate [1, 2]. Previous studies have documented an association between short LTLs and increased risk of early death as well as cardiovascular disease, type 2 diabetes mellitus, and cancer [3–7]. In contrast, increases in LTL have been found to be associated with an increase in telomerase activity, which can occur in response to positive lifestyle changes and stress reduction [8–10]. Short-term changes in LTLs, even over an interval as short as 9 months similar to term gestation, have been found to be related to changes in adult brain structure [11]. Given the physical, biochemical, and psychological stressors of pregnancy, the clinical implications of LTL shortening in non-pregnant adults, and correlation between short-term changes in LTL and physiologic changes in humans, it is possible that maternal LTL is affected – as either a contributor or a consequence – by human gestation. As such, it is important to know the natural history of gestational telomere dynamics to inform future research utilizing this biomarker in pregnancy.

The likely importance of telomeres during pregnancy has been described [12]. However, previous studies were limited to animal models [13, 14], and human studies either lack granularity in pregnancy characteristics, were cross-sectional, or focused primarily on placental or offspring telomeres [2, 15–18]. Given the biochemical changes during pregnancy, the postulated role of inflammation in contributing to adverse perinatal events such as preeclampsia and preterm birth [19], and the relationship between telomere shortening and inflammatory processes such as oxidative stress [20], it is important to understand whether pregnancy affects natural telomere dynamics. To this end, we characterized LTL changes during pregnancy and in the early postpartum period in a pilot study using a cohort of healthy participants with uncomplicated, term pregnancies. In addition, we examined demographic characteristics, self-reported perceived stress and lifestyle habits, and postpartum depression scores among the cohort to contextualize LTL findings.

## Methods

### Study design

Pregnant participants who had been enrolled in a longitudinal study conducted by the March of Dimes Prematurity Research Center at Stanford University between 2012 and 2018 and who presented for obstetric care prior to 12 weeks of gestation at Stanford University Hospital and Clinics were included in this pilot study. Participants provided responses to a survey and provided biological samples during pregnancy and the early postpartum period; the details of this survey have been previously described [21]. The objective of our present study was to utilize this cohort to characterize LTL dynamics in participants with uncomplicated pregnancies in order to provide pilot data for future research on populations with pregnancy complications. Therefore, we included only nulliparous participants with singleton livebirths at or beyond 37 weeks of gestation using the best obstetric estimate determined by the participant’s provider. Because the purpose of this study was to estimate the effect of an uncomplicated pregnancy on maternal LTLs, participants were excluded if they had diabetes mellitus (preexisting or gestational) or developed preeclampsia during pregnancy. Longitudinal blood samples were collected from each person over the course of pregnancy and the early postpartum period, plasma was separated and further processed for isolation of peripheral blood mononuclear cells (PBMCs). Peripheral blood mononuclear cells (PBMCs) were prepared and cryopreserved according to standard protocols. BD Vacutainer CPT Cell Preparation Tubes with Sodium Citrate (CPT) were used for collection. All samples were then immediately stored at − 80 °C until analyses. All patients had at least one stored blood sample collected during their pregnancy or early postpartum.

Blood samples were collected during one of three time periods: prior to 20^0/7^ weeks of gestation (Timepoint 1); between 20^1/7^ and 36^6/7^ weeks of gestation (Timepoint 2); or between 37^0/7^ weeks of gestation and 9-weeks postpartum (Timepoint 3), as pregnancy physiology can persist up to 12 weeks after delivery [22]. For reference, weeks of gestation were defined as the completed number of weeks and number of additional days out of 7 beyond this as superscript; for example, a subject who was 35 weeks and 5 days pregnant was listed as being 35^5/7^ weeks gestation. This study was approved by the Institutional Review Board at Stanford University (Protocol Number 21956). During enrollment, written informed consent was obtained from all patients for participation in the study as well as for future research using archived samples and medical records.

### LTL measurements

LTLs were measured according to previously published protocols, specifically the method described by Cawthon et al. [23, 24]. Frozen PBMCs were thawed at room temperature for 20 min and centrifuged at 7000 rpm for 5 min at 4 °C. Cell pellets were resuspended and genomic DNA extracted using the QIAamp protocol for cultured cells [25]. As per this previously published protocol [23], telomeric (“T”) and single copy gene (human beta globin, “S”) values for each sample were determined by quantitative polymerase chain reaction (qPCR) using Roche LC480 real-time PCR machine (Roche Diagnostics Corporation, Indianapolis, IN). The cycling protocol for T PCR was as follows: denature at 96 °C for 1 min, denature at 96 °C for 1 s, anneal/extend at 54 °C for 30 s with fluorescence data collection for 30 cycles, 95 °C for 30 s with continuous fluorescence data collection during the rise to 95 °C. The cycling protocol for S PCR was as follows: denature at 94 °C for 1 min, denature at 95 °C for 15 s, anneal at 58 °C for 1 s, extend at 72 °C for 20 s for 8 cycles without data collection, denature at 96 °C for 1 s, anneal at 58 °C for 1 s, extend at 72 °C for 20 s, hold at 83 °C for 7 s with single fluorescence data collection for 34 cycles, and lastly melt at 95 °C for 1 min, anneal at 54 °C for 30 s, 95 °C for 30 s with continuous fluorescence data collection during the rise to 95 °C.

In this previously published protocol [23, 24], the primers for the telomere PCR are *tel1b* [5′-CGGTTT (GTTTGG)_5_GTT-3′] at a final concentration of 100 nM and *tel2b* [5′-GGCTTG (CCTTAC)_5_CCT-3′] at 900 nM. The primers for the single-copy gene (human beta-globin) PCR were *hbg1* [5′ GCTTCTGACACAACTGTGTTCACTAGC-3′] at a final concentration of 300 nM and *hbg2* [5′-CACCAACTTCATCCACGTTCACC-3′] at 700 nM. The final reaction mix contained 20 mM Tris-HCl, pH 8.4; 50 mM KCl; 200 μM each of A, C, G and T dNTP; 1% DMSO; 0.4x Syber Green I; 22 ng *E. coli* DNA; 0.4 Units of Platinum Taq DNA polymerase (Invitrogen Inc.); approximately 6.6 ng of genomic DNA per 11 μL reaction. Tubes containing 26, 8.75, 2.9, 0.97, 0.324, and 0.108 ng of a reference DNA (human genomic DNA from buffy coat, Sigma-Aldrich, Cat#11691112001) were included in each PCR run to determine the quantity of targeted templates in each research sample relative to the reference DNA sample using a standard curve. The same reference DNA was used for all PCR runs. Assays were run in triplicate wells on 384-well assay plates in a Roche LightCycler 480. The average concentrations of T and S were used to calculate T/S ratios after a Dixon’s Q test to remove outliner wells from the triplicates. T/S ratio for each sample was measured twice. When the duplicate T/S values and the initial value varied by more than 7%, the sample was run the third time and the two closest values were reported. To adjust for batch effect, each run included the same 8 control DNA samples (run in 6 wells on the 384 plate) and the T/S ratios of these control DNAs were compared with the mean of the first 10 runs of this batch of control samples to obtain an adjustment factor for each sample. The mean of the 8 adjustment factors was applied to the testing samples to convert the raw to adjusted T/S ratios. Adjusted T/S ratios were used in further analyses.

### LTL changes during pregnancy

First, the mean LTL for all patients was determined at each timepoint for which they had usable data. Next, the mean change in LTL between timepoints within an individual for those with logitudinal LTL measurements was calculated in order to determine the change per individual between Timepoints 1 and 2, Timepoints 2 and 3, and Timepoints 1 and 3. Using this approach, the difference in LTL between Timepoints 1 and 3 would approximate the difference in LTL across the pregnancy from the late first trimester into the postpartum period. Given the possible impact of post-operative inflammatory physiology on telomere length, we also compared LTLs as a function of mode of delivery (vaginal versus cesarean) in a subgroup analysis with participants with postpartum LTLs from Timepoint 3.

### Perceived stress assessment

During enrollment in the first trimester, demographic information was recorded by both self-report and chart review; this information included race/ethnicity, educational attainment, weight, and height. In addition, participants responded to questionnaires assessing several psychosocial stress indicators. Some examples of the stress indicators included questions to assess perceived risks to the pregnancy (e.g., “my risk of birth complications is higher than other pregnant patients of similar age”), exercise during pregnancy, degree of stress during different periods of life including the year prior to pregnancy, and sleep quality. Edinburgh Postpartum Depression Scale (EPDS) scores were obtained at the 6-week postpartum visits and recorded if available.

Responses to the psychosocial stress indicator surveys (hereafter referred to as “features”) were correlated with LTL using machine-learning analysis. This was done to evaluate associations between individual stress features and LTLs at Timepoint 1 as well as mean LTL across all timepoints. We analyzed 79 features related to specific questions on the survey using a previously published approach [21]. First univariate associations between stress features and both Timepoint 1 and mean LTLs were investigated using appropriate tests for numeric (Kendals Tau), categorical (Kruskal) and binary variables (Wilcoxon rank-sum). To visualize the relation between stress features together with their association to LTLs, we drew a correlation plot network, first imputing missing values with medians, then calculating the correlation matrix of all features, and then applying t-distributed Stochastic Neighbor Embedding (t-SNE) [26] on the absolute values of the matrix to derive feature coordinates in two-dimensional space. Node sizes represent the strength of association of each feature with LTL measured by the corresponding *p*-value. In an attempt to determine whether the stress measures collectively could predict LTL, a support vector machine was trained to predict LTLs from the multi-variate stress profile and evaluated using 10-fold cross-validation.

### Statistical analyses

First, means and standard deviations were calculated for LTLs at each timepoint for all available samples. Next, LTL changes within patients between timepoints were assessed using the Wilcoxon signed-rank test. Given our small sample size, we did not adjust for potential confounders. For the subgroup analysis, we compared postpartum LTLs between those with vaginal versus those with cesarean births using Wilcoxon rank sum given that LTLs were not normally distributed. Additional adjustment for maternal age was done using linear regression modeling after log transformation of LTL and confirmation of linearity in association between maternal age and log (postpartum LTL). Responses to the stress indicator survey and EPDS scores were reported descriptively for participants who had LTL results from both Timepoint 1 and 3 across pregnancy, then graphically for the machine learning analysis data. STATA version 16 (College Station, TX) was used for statistical analysis and common statistical and machine learning Python libraries were used including “Scitkit-Learn” and “statsmodels” (in Python 3.7). Statistical significance was set a priori for all tests at two-sided alpha = 0.05.

## Results

A total of 46 participants with 115 blood samples comprised our study cohort (Fig. 1). The mean age of these 46 participants was 29.8 ± 3.8 years and mean enrollment body mass index (BMI) was 21.7 ± 2.8 kg/m^2^. The majority of participants were privately insured (91.3%) and had completed a college degree or higher (87.8%, Table 1). 18 (39.1%) patients underwent a cesarean birth. Among these, the most common indications were labor arrest (38.9%), breech presentation (27.8%), and fetal intolerance of labor (22.2%).

**Fig. 1:** Consort Diagram

**Table 1:** Demographics and perinatal outcomes for our study cohort of nulliparous patients with term, singleton livebirths between 2012 and 2018

Characteristic or Outcome	Whole cohort *n* = 46^a^	Participants with both Timepoints 1 and 3 leukocyte telomere lengths (LTL) *n* = 32
Mean age at enrollment (years)	29.8 ± 3.8	30.1 ± 3.9
Mean BMI at enrollment (kg/m^2^)	21.7 ± 2.8	22.1 ± 2.8
Race/Ethnicity		
Asian	7 (15.6%)	6 (18.8%)
Hispanic	6 (13.3%)	3 (9.4%)
Indian	3 (6.7%)	2 (6.3%)
White	26 (57.8%)	19 (59.4%)
Multi-race	3 (6.7%)	2 (6.3%)
Private insurance	42 (91.3%)	29 (90.6%)
Completed college or higher degree	36 (87.8%)	24 (85.7%)
Spontaneous conception	41 (89.1%)	28 (87.5%)
Mean gestational age at delivery (weeks)	39.1 ± 1.3	39.2 ± 1.3
Cesarean birth	18 (39.1%)	13 (40.6%)
Mean neonatal birthweight (g)	3335 ± 411	3361 ± 466

^a^Mean ± SD shown for continuous variables, n (%) shown for categorical variables. Percentages exclude missing data, which included 1 (2.2%) missing race/ethnicity, 5 (10.9%) missing BMI, 5 (10.9%) missing education, and 1 (2.2%) missing birthweight

The coefficient of variation (CV) for LTL measurements was 2.2%. The PCR efficiencies of the telomere (T) and single-copy (S) gene reactions for this study were 93.2 ± 4.2% and 94.0 ± 4.2%, respectively. Mean LTLs for each timepoint are presented for the whole cohort (*n* = 46) and for the subset with LTL results from both Timepoints 1 and 3, shown to illustrate change over the course of pregnancy (*n* = 32, Table 2). LTL changes across gestation are shown graphically in Fig. 2 and individual panel graphs for LTL across gestation for each patient are shown in Fig. 3. Note that gestational ages (GA) were reported as weeks since last menstrual period, so samples collected postpartum were recorded as up to 50 weeks of gestation for a common time scale. For the 35 participants with Timepoint 3 LTLs, the vast majority of samples (*n* = 32, 91.4%) were collected postpartum.

**Table 2:** Telomere dynamics across gestation for nulliparous patients with term, singleton livebirths between 2012 and 2018

Characteristic	Whole cohort *n* = 46^a^	Cohort with Timepoint 1 and Timepoint 3 *n* = 32^a^
Mean first LTL (T/S)^b^	1.15 ± 0.26	1.12 ± 0.22
Mean second LTL (T/S)^c^	1.13 ± 0.23	1.14 ± 0.26
Mean third LTL (T/S)^d^	1.07 ± 0.21	1.05 ± 0.20
Mean gestational age (GA) at Timepoint 1 (weeks)	12.0 ± 2.6	11.9 ± 2.6
Mean GA at Timepoint 2 (weeks)	26.5 ± 1.8	26.4 ± 1.8
Mean GA at Timepoint 3 (weeks)	42.8 ± 3.0	43.1 ± 2.9

^a^Mean ± SD shown

^b^First sample collected before 20^0/7^ weeks, *n* = 41

^c^Second sample collected between 20^0/7^ and 36^6/7^ weeks, *n* = 39

^d^Third sample collected between 37^0/7^ weeks of pregnancy and up to 9-weeks postpartum, *n* = 35

**Fig. 2:** Leukocyte telomere length (LTL) by week of gestation among nulliparous patients with term, singleton livebirths from 2012 to 2018

**Fig. 3:** Maternal leukocyte telomere length dynamics (T/S ratios) by gestational age (GA) for each study participant, *n* = 46

LTLs reported as T/S ratios for each sample collected. Of 41 samples collected before 20 weeks, mean T/S ratio was 1.15 ± 0.26; of 39 samples collected between 20^0/7^ and 36^6/7^weeks, mean T/S ratio was 1.13 ± 0.23; of 35 samples collected after 37^0/7^ weeks, mean T/S ratio was 1.07 ± 0.21. Samples collected postpartum are recorded as up to 50 weeks of gestation for a common time scale. Loess smooth line applied to demonstrate trend across scatter plot, which was non-significant.

Maternal LTL T/S ratios shown on y-axis and GA on x-axis for each participant to demonstrate individual changes in LTL during pregnancy using longitudinal measurements. Graphs that appear to be blank have only one LTL measurement available; therefore, a line between points was not possible. Lines with a positive slope correspond to LTL increases; lines with a negative slope indicate LTL decreases.

Among participants with multiple LTL timepoint results, there were no significant differences in within person LTL between any timepoints. Specifically, there was no difference between Timepoints 1 and 2 (T/S difference: − 0.03 ± 0.26, *p* = 0.39), Timepoints 2 and 3 (T/S difference: − 0.07 ± 0.29, *p* = 0.38), or Timepoints 1 and 3 (− 0.07 ± 0.2, *p* = 0.06). When comparing postpartum LTL by mode of delivery, participants who underwent cesarean birth had significantly shorter LTL than did those who delivered vaginally (T/S ratio: 0.94 ± 0.12 cesarean versus 1.12 ± 0.21 vaginal, *p* = 0.01, Fig. 4). In multivariable linear regression modeling accounting for maternal age, the association between cesarean and shorter postpartum leukocyte telomere length persisted (beta − 0.18, 95% CI − 0.30 to − 0.05, *p* = 0.006). It is important to note that there was no significant difference in when the postpartum draw for LTL occurred between cesarean versus vaginal births (mean ± SD 43.5 ± 2.8 weeks for cesarean versus 42.9 ± 3.1 weeks for vaginal, Wilcoxon rank-sum *p* = 0.47).

**Fig. 4:** Postpartum maternal leukocyte telomere length (LTL) shorter after cesarean compared with vaginal deliveries (*n* = 32)

Box plots of postpartum leukocyte telomere length compared between participants with vaginal versus cesarean births using Wilcoxon rank sum test (mean ± SD 0.94 ± 0.12 cesarean versus 1.12 ± 0.21 vaginal, *p* = 0.01).

Next, we conducted our secondary analysis evaluating EPDS scores and stress surveys. The mean EPDS score for the cohort was 4.4 ± 3.3; only 2 (9.5%) of participants in the cohort had a positive EPDS screen with a score of 10 or higher. Stress-indicator survey responses were available for 32 patients with both Timepoint 1 and 3 LTL measurements, although not all surveys were complete (Table 3). Completeness ranged from 87.5 to 100% among individual questions. Notably, only 13.8% of patients had reported that the preceding year had been very stressful for them.

**Table 3:** Perceived stress survey responses and telomere dynamics among healthy, nulliparous patients with term livebirths with leukocyte telomere length (LTL) results from the beginning of pregnancy and delivery/postpartum from 2012 to 2018

Survey Response	Cohort with LTL results from Timepoints 1 and 3 *n* = 32^a^ N (%)
Perceived risk of birth complications higher than other pregnant women of similar age (*n* = 32)	7 (21.9)
Perceived risk of birth defects higher than other pregnant women (*n* = 31)	6 (19.4)
Current vigorous physical exercise during pregnancy (*n* = 31)	3 (9.7)
Current moderate physical exercise during pregnancy (*n* = 32)	21 (65.6)
Amount of moderate exercise less than prior to pregnancy (*n* = 21)	8 (3.8)
The past year has been very stressful (score 6 to 7) (*n* = 29)	4 (13.8)
Stressful or very stressful first 10 years of age (*n* = 29)	2 (6.9)
Stressful or very stressful 11 to 20 years of age (*n* = 29)	4 (13.8)
Stressful or very stressful 21 to 30 years of age (*n* = 28)	4 (14.3)
Experienced death of a loved one (*n* = 29)	21 (7.2)
Poor to very poor sleep on weeknights (*n* = 29)	1 (3.4)
Frequent episodes of pain (e.g., headaches, backaches, soreness, etc) (score 6 to 7) (*n* = 29)	3 (10.3)
Sad feelings for the last 3 years (*n* = 29)	1 (3.4)
Happy or very happy feelings the last 3 years (*n* = 28)	21 (75.0)
Edinburgh Postpartum Depression Scale (EPDS) score (*n* = 21)	4.4 ± 3.3

^a^Categorical values listed as n (%) or mean ± SD

Twenty-seven participants had complete data available for inclusion in the machine learning analysis that focused on domains of stress features within the surveys. Because there were no significant differences in LTL across gestation as described above, we used Timepoint 1 LTL and mean LTL values for this analysis because we felt that a single LTL measure, rather than a difference between LTL measures, better captured potential associations and reduced variability in results. This was because a single LTL measure rather than a difference between LTL measures was felt to better capture potential associations and reduce variability in results. We identified stress measures, including lower assessment of current health (*p* = 0.02) and poor sleep quality (p = 0.02), which were associated with shorter Timepoint 1 LTL (not corrected for multiple comparisons, Fig. 5). When LTLs were averaged across all available timepoints for each participant, poor sleep quality remained significantly associated with shorter LTL (*p* = 0.03). The trained model to predict LTL (first timepoint or mean) from the multi-variate stress profile did not yield significant predictive power for overall stress and LTL.

**Fig. 5:** Correlation network visualizing the univariate analysis of stress features and Timepoint 1 LTL

Nodes are colored if *p* < 0.1. Node labels are bold, if *p*-values pass the *p* < 0.05 threshold. For these thresholds, no multiple comparison adjustment was performed. Node colors represent positive (orange) and negative (blue) associations with LTL. Edges represent Spearman correlations between stress variables. Thin edges represent absolute correlation with *r* > = 0.3 while thick edges represent an absolute correlation of *r* > = 0.7.

## Discussion

In this pilot study, we reported longitudinal LTL measurements across gestation in 46 nulliparous patients with uncomplicated, term pregnancies. There were no significant differences in maternal LTLs over the course of gestation in this cohort, which also had a low prevalence of stress and depression as indicated by survey responses and EPDS scores. Furthermore, our assessment of maternal LTLs and perceived stress revealed poor sleep quality to be associated with maternal LTL at Timepoint 1 and when averaged across all timepoints. With respect to mode of delivery, participants who underwent cesarean birth had shorter postpartum LTL than did those who had a vaginal birth. These results can inform future research on LTLs as a biomarker in pregnancy; leukocyte telomere length sampling at any single timepoint in pregnancy is likely adequate, but if sampling is done postpartum consideration should be made regarding the effect of mode of delivery. While these observations provide groundwork for future investigations, their validation, and particularly the underlying causal dependencies, require examination in larger datasets.

In the context of this biologically plausible connection, there have been conflicting data concerning whether pregnancy affects the rate of maternal LTL shortening [27–32]. While the average LTL shortening in non-pregnant adults has been reported to range from 10 to 50 bp in 1 year, one large cross-sectional study by Pollack *et. al*. [31] demonstrated that LTL in 1954 parous participants was, on average, 116 bp shorter than it was in nulliparous participants after adjusting for multiple confounders, including age. Their large sample size provided ample power to evaluate small differences in LTL by parity, which was more limited in our study; however, this study did inform our decision to restrict the cohort only to nulliparas.

In contrast, other studies – including ours – have not found a significant reduction in LTLs during pregnancy. It may be that the immunotolerant state of pregnancy attenuates the expected telomere shortening, or, as above, that the postpartum period (rather than the pregnancy) affects LTL shortening. It is also possible that heterogeneity in risk profiles of pregnancies included in prior studies obscured LTL changes [15, 33]. In this context, we specifically excluded high-risk pregnancies from our cohort in order to ascertain the natural history of maternal telomere dynamics in a low risk population. Even after doing so, we still identified both LTL shortening and LTL lengthening, which may have attenuated the overall LTL change toward the null.

The phenomenon of increasing LTLs has been previously described and may be related to the upregulation of telomerase, decreases in shelterin protein activity – which protects telomeres from pathologic lengthening – or even changes in the leukocyte composition of a sample [30, 34, 35]. Furthermore, variability in LTL has been established even within leukocyte subclasses outside of pregnancy [36]. Whether the increases in LTLs we identified points to variabilities in our measurements of LTLs, a regression to the mean phenomenon – where natural variation in longitudinal biologic measurements can result in repeat values being closer to the true mean value [37] – or highlights the complexity of the underlying mechanism remains to be elucidated in a larger cohort.

It is also important to note that postpartum LTLs were significantly shorter in participants who underwent cesarean vs. vaginal delivery. The average timing of LTL sample collection was on average more than 1 week postpartum, when patients would likely be outside the immediate post-operative inflammatory window during which a leukocytosis could affect LTLs. While data are lacking concerning the post-operative inflammatory response following cesarean, high levels of pro-inflammatory cytokines have been reported at 48 h after abdominal hysterectomy which may serve as a surgical correlate for cesarean [38]. Given the known relation between LTL shortening and inflammation, it is possible that the shorter LTLs seen in this group reflect the post-operative state. Further investigation in this area is warranted given that there are limited data concerning how surgery might affect LTL. At the very least, this highlights the importance of consideration of mode of delivery in future studies investigating telomere length change in pregnancy, specifically when evaluating LTLs collected postpartum.

Our secondary analysis highlighted poor sleep quality as a stress measure associated with shorter maternal LTLs. Studies outside of pregnancy have also reported a significant association between poor sleep and short LTLs [39, 40]. While data on maternal LTL and sleep are limited, researchers have examined the association between maternal sleep in pregnancy and neonatal LTL, with conflicting results [41]. Based on our results, a more focused evaluation of sleep and maternal LTL is warranted.

We note important limitations of our study. First, our small sample size, while comparable to other studies of telomeres, limited our power and ability to explore population subgroups or adjust for potential confounders. As a related point, our sample included only healthy pregnancies; future research should extend our findings to more complex pregnancies. Second, there was some variability in timing of maternal blood sample collection, which was most notable for Timepoint 3 with a standard deviation of 2 to 3 weeks. We were also unable to control for time of day at blood draw which may have increased variability of our results. While the CV was small among the LTL measurements, it is possible that some small differences in LTLs for some participants represent error or variance of the assay; future research with larger cohorts would help address this question. Additionally, the demographic makeup of our cohort encompassing highly educated and insured participants may limit the external generalizability of our findings but does provide internal validity. Research investigating telomere dynamics in pregnancy in more diverse cohorts is warranted.

The strengths of this study included our ability to compare longitudinal LTL measurements within one pregnancy. By reporting mean T/S ratios across gestation in a healthy cohort with uncomplicated pregnancies, we have characterized baseline LTL dynamics in normal pregnancies. Specifically, these baseline data may be used to help design future research in this area. In addition, our machine learning analysis provides a complementary, rigorous comparison between biologic and psychological stress measures that aids in interpretation of our results.

## Conclusions

In conclusion, our results provide valuable baseline information suggesting that LTL does not change significantly over the course of healthy pregnancies; this information can inform directions for future research on this topic. Prospective research with a larger, more diverse cohort is warranted. Correlating LTLs with known inflammatory markers and white blood cell counts during pregnancy may further illuminate on our results, but this was beyond the scope of the current study and is an ongoing area of future research.

Given the biochemical, physical, and psychologic stressors of pregnancy, we hypothesized that significant LTL shortening would have been identified for all participants in this cohort. Although there were trends toward overall LTL shortening, we did not identify significant changes in LTLs over the course of gestation. Whether this is due to the low prevalence of stress in this cohort, the variability in LTL measurements, or is a true biologic phenomenon remains to be elucidated. Our results underscore the importance of accounting for mode of delivery when studying postpartum LTL, as participants who underwent cesarean had shorter postpartum LTLs compared with those who had a vaginal birth. Finally, we identified an association between poor sleep quality and shorter LTLs which may direct future work in this area.

## Supplementary Information

**Additional file 1.**

## Data Availability

Deidentified datasets used during the current study are uploaded as supplemental files. The machine learning analysis is available on request to the corresponding author.

## Abbreviations

bp: Basepairs
CV: Coefficient of variation
EPDS: Edinburgh Postpartum Depression Scale
LTL: Leukocyte telomere length
GA: Gestational age
PBMCs: Peripheral blood mononuclear cells
T/S ratio: Telomere to single copy gene ratio
